# TDP-43 causes neurotoxicity and cytoskeletal dysfunction in primary cortical neurons

**DOI:** 10.1371/journal.pone.0196528

**Published:** 2018-05-22

**Authors:** Pranetha Baskaran, Christopher Shaw, Sarah Guthrie

**Affiliations:** 1 Department of Developmental Neurobiology, King's College, Guy's Campus, London, United Kingdom; 2 Maurice Wohl Clinical Neuroscience Institute, King's College, London, United Kingdom; International Centre for Genetic Engineering and Biotechnology, ITALY

## Abstract

TDP-43-mediated proteinopathy is a key factor in the pathology of amyotrophic lateral sclerosis (ALS). A potential underlying mechanism is dysregulation of the cytoskeleton. Here we investigate the effects of expressing TDP-43 wild-type and M337V and Q331K mutant isoforms on cytoskeletal integrity and function, using rat cortical neurons in vitro. We find that TDP-43 protein becomes mislocalised in axons over 24–72 hours in culture, with protein aggregation occurring at later timepoints (144 hours). Quantitation of cell viability showed toxicity of both wild-type and mutant constructs which increased over time, especially of the Q331K mutant isoform. Analysis of the effects of TDP-43 on axonal integrity showed that TDP-43-transfected neurons had shorter axons than control cells, and that growth cone sizes were smaller. Axonal transport dynamics were also impaired by transfection with TDP-43 constructs. Taken together these data show that TDP-43 mislocalisation into axons precedes cell death in cortical neurons, and that cytoskeletal structure and function is impaired by expression of either TDP-43 wild-type or mutant constructs in vitro. These data suggest that dysregulation of cytoskeletal and neuronal integrity is an important mechanism for TDP-43-mediated proteinopathy.

## Introduction

It is well established that mutations of the TAR DNA-binding protein 43 (TDP-43), a highly conserved nuclear protein, are causal of Amyotrophic Lateral Sclerosis (ALS), and in the most common variant of Frontotemporal Lobe Dementia, FTLD-U [1–4]. Several groups have identified mutations in TDP-43 in sporadic and familial cases of ALS and have provided evidence of a direct link between TDP-43 dysfunction and neurodegeneration[3–5]. Previous studies in transgenic animal models have shown that over-expression of wild-type and mutant isoforms of TDP-43 is toxic and can cause neurodegeneration.

TDP-43 is predominantly a nuclear protein, although it is actively shuttled between the nucleus and the cytoplasm [6] However, under pathological conditions, TDP-43 is depleted from the nucleus and accumulates in the cytoplasm in both neurons and glia [7, 8]. Thus TDP-43 proteinopathies could be caused by a loss of function due to nuclear depletion, by a gain of function due to cytoplasmic aggregation, or by a combination of both [1, 9–11]. Pathological TDP-43 is abnormally ubiquitinated, hyperphosphorylated and N-terminally cleaved to generate C-terminal fragments (20–25 kDa) [12]. The fundamental question as to whether TDP-43 mediates neurodegeneration via a gain of function or a loss of function remains unanswered.

TDP-43 is an RNA binding protein which plays an important role in mRNA transport, stability, and translation [13, 14]. TDP-43 directly interacts with the 3’UTR of neurofilament light chain (68 kDa) mRNA to stabilise it [15], and associates with *futsch* (MAP1B) mRNA in a complex *in vivo* to regulates its localization and translation in *Drosophila* motor neurons [16]. Hence, a plausible hypothesis is that TDP-43 brings about neuronal death by dysregulation of cytoskeletal components [17]. TDP-43 has been shown to play a role in the regulation of axon growth and in axonal transport [6, 18].

Most studies have used transgenic animals and cell lines to investigate TDP-43 pathomechanisms with fewer studies on primary neurons [6, 19, 20]. We have previously shown that in chick spinal motor neurons and *in vitro* and *in vivo*, TDP-43 mis-localises in axons, coinciding with a reduction in axonal length and an increase in cellular toxicity [21]. In the present study, primary cortical neurons are a relevant cell type due to the involvement of TDP-43 in FTLD-U, which affects cortical neurons.

Here we compare the effects of transfecting into rat cortical neurons wild-type TDP-43, and two mutant isoforms containing the M337V familial mutation or the Q331K sporadic mutation. Both are missense mutations in the highly conserved glycine-rich C-terminus of TDP-43 which mediates protein-protein interactions [4]. These two mutants were shown to provoke age-dependent, progressive motor neuron degeneration when expressed in mice at levels similar to endogenous TDP-43 [22]. We have previously shown that both TDP-43 mutant isoforms also cause apoptosis in the chick spinal cord, suggesting a toxic gain of function or dominant-negative effect [4]. The effects of TDP-43 overexpression on toxicity, the localisation of TDP-43 protein, axonal growth, cytoskeletal integrity and axonal transport were analysed using toxicity assays, immunohistochemistry and live imaging.

## Materials and methods

### Plasmids

The GFP-tagged *WT-TDP-43*, *M337V-TDP-43* and *Q331K-TDP-43* constructs and *GFP* control plasmids were as described previously [21]. The *EB3-RFP* construct was a gift from Maddy Parsons’s lab (Randall Division of Cell & Molecular Biophysics).

### Primary rat cortical neuron cultures and transfection

Sprague-Dawley rats pregnant with E18 embryos were obtained from Charles River UK, Ltd., located in Manston Road. Margate CT9 4LT. The animals were bred for research purposes. E18 rat cortices were dissected in ice-cold Hanks Buffered Salt Solution (HBSS; Invitrogen), equilibrated for 2 minutes, and incubated with trypsin diluted 1:4 in HBSS for 15 mins at 37°C with intermittent shaking for 15 mins. Trypsin inhibitor solution was then added and the cortices were dissociated by trituration and centrifuged for 5 mins at 1200 rpm. The supernatant was removed, the pellet was re-suspended in 5 ml of pre-warmed HBSS, passed through a 70 µm filter and re-centrifuged as above. The pellet was resuspended in 2ml of pre-warmed HBSS and the number of cells was counted using a haemocytometer. For non-transfected cells, 80,000 cells from the cell suspension was centrifuged at 1800 rpm for 5 mins and the pellet was re-suspended in 400 µl of culture medium per well.

For transfection, the required number of cells (4–5 x 10^6^ cells per plasmid construct) to be transfected was centrifuged at 1800 rpm for 5 mins. The neurons were transfected using an Amaxa machine with rat neuron nucleofector solution (Lonza). The cell pellet was resuspended in 100 µl of nucleofector solution with 4 µg of DNA, transferred into the Amaxa cuvette and transfected using the O-003 program. 200 µl of pre-equilibrated culture medium was added and cells were plated at a density of 100,000 cells in 400 µl of culture medium per well. Transfection efficiency was ~70%.

Neurons were cultured on 13 mm round coverslips that had previously been coated with poly-lysine and laminin (Sigma-Aldrich) in multiwell plates (Nunc). Confocal dishes (Ibidi) were used for live imaging. The culture medium was Neurobasal with 2% B-27, 1% glutamax and 1% penicillin-streptomycin (all from Invitrogen) with 2% horse serum (Sigma-Aldrich). Cultures were incubated at 37°C with 5% CO_2_ for 24–120 h. For cultures that were maintained for < 48 h, the medium was replaced every two days.

### Immunocytochemistry

Primary antibodies used were chick anti-GFP (1:1000; Abcam), rabbit anti-TDP43 (1:1000; Cell Signalling), rabbit anti-neurofilament-H (1:1000; Millipore), rat anti-tyrosinated tubulin (1:1000; Abcam) and rabbit anti-Glu-tubulin (1:1000; Abcam). Secondary antibodies were anti-rabbit Cy-3-conjugated, anti-chick Alexafluor488, anti-rabbit Alexafluor 568 and anti-rat Alexafluor 568 (all at 1:1000; Life Technologies).

Coverslips were fixed by adding 400 µl of 4% paraformaldehyde (PFA)/15% sucrose (Sigma-Aldrich) to each well for 15 mins at room temp, then washed twice with PBS-T (1 X phosphate-buffered saline (PBS) + 0.1% Triton X-100) and rocking. Non-specific binding was blocked using 0.5% bovine serum albumin (BSA; Sigma) in PBS for 1 h at room temp. Coverslips were incubated in primary antibodies diluted as above in 0.1% PBS-T with 0.5% FBS, overnight on a rocker at 4°C, then washed 3 X 10 mins with PBS-T on a rocker plate at room temperature, followed by incubation in secondary antibodies as above in PBS-T for 1–2 h at room temperature with rocking. After further washes, the coverslips were mounted on slides using Fluorsave (Calbiochem) with Hoechst reagent (Thermo-Fisher Scientific).

### TUNEL toxicity assay

Terminal Deoxynucleotidyl Transferase dUTP Nick End Labeling (TUNEL) was used to detect fragmented DNA associated with cell apoptosis, using the DeadEnd colorimetric TUNEL system (Promega) according to the manufacturer's instructions. Before starting the assay, cells were permeabilised for 5 mins with 100 µl of 20 µg/ml of Proteinase K in PBS-T. Coverslips were washed twice with PBS-T with 2 mg/ml of glycine, then fixed for 5 mins with 4% PFA, and washed twice with PBS-T. After the diaminobenzidine staining step of the assay, coverslips were washed several times with water, fixed with 4% PFA for 10 mins and immunostained with the respective primary and secondary antibodies as above.

The TUNEL-positive cells appeared as black dots and were manually counted from five different 0.24 mm^2^ fields from a 13 mm coverslip. A comparison with the Hoechst nuclear staining (Invitrogen) using blue epifluorescence gave the total cell numbers. Three coverslips from three experiments per condition was used to average the number of TUNEL-positive cells.

### Cell viability assay

Cortical neuron cultures were plated on white opaque-walled 96 well plates. Cell viability was monitored using a continuous read format with the Promega RealTime-Glo™ MT Cell Viability Assay. The MT Cell Viability Substrate and NanoLuc® Enzyme were added to the culture medium at the dosage specified by the protocol, plates were re-incubated for 4 h and the first luminescence reading was taken 24 h after transfection and every 24 h thereafter using a luminescent plate reader. The average relative light unit (RLU) from three different experiments, as measured by the luminometer, was plotted for the different constructs against the different time-points.

### Live imaging of cortical neurons

For live imaging, neurons were plated on confocal dishes at a density of 160,000 cells per well in 1 ml of medium. For EB3 imaging, rat cortical neurons were co-transfected with equal quantities of the GFP control plasmid or TDP-43 wild-type and mutant plasmids together with an RFP-tagged EB3 plasmid. Neurons were imaged in a Nikon Live imaging chamber microscope maintained at 37°C with 5% CO_2_. Transfected neurons that expressed GFP were imaged at 60X with the DIC channel for 30 mins with 2–5 sec intervals using Nikon Elements software.

### Axon length and growth cone analysis

For axon length measurements, the length of 100 neurons per transfection per experiment (n = 3) were measured using neuron J, selecting healthy neurons with an uninterrupted axon that was at least 3 times the length of the cell body.

The growth cones of neurons labelled with anti-GFP and anti-tubulin antibodies were imaged using a Zeiss AxioScop at 63X, and images were processed using Volocity or ImageJ software. ImageJ was used to quantitate growth cone area, by thresholding the GFP fluorescence, drawing an outline and measuring the area in pixels. A total of ~70 neurons per construct were analysed from 3 independent experiments. The graphs were drawn based on the average area and Standard error of mean.

### Kymographs

To quantitate EB3 ‘comet’ velocities along axons, we used kymographs, made using ImageJ and analysed using Kymoquant^TM^ software, which calculates the velocity of individual EB3 traces based on the angle and tangent of the kymograph patterns. A total of 20 movies from 3 independent experiments were analysed. The graphs were drawn based on the average velocity in pixels/frame and standard error of mean. Kymographs were drawn for 10 neurons per construct per experiment (n = 3) using Image J.

### Statistics

Statistics used a one-way Anova coupled with Dunn's multiple comparison test.

### Ethics

The research was approved by the Home Office UK and the ethics committee of Kings College London—College Research Ethics Committee (CREC). The Project was reviewed by the Biomedical Sciences, Medicine, Dentistry and Natural & Mathematical Sciences Research Ethics Sub-Committee (BDM RESC). The rats used in the experiments were humanely killed by cervical dislocation, under the “Schedule 1 to the animals (Scientific Procedure) Act 1986”.

## Results

### TDP-43 is mislocalised and aggregated in cortical neurons

TDP-43 protein aggregation and mislocalisation is a hallmark of ALS. We have previously shown that TDP-43 shows enhanced cytoplasmic mislocalisation over time in chick spinal motor neurons and in the spinal cord *in vivo* [21]. Given that TDP-43 pathology also occurs in FTLD-U, which affects the cortex, we determined whether cortical neurons in vitro have the same vulnerability as spinal motor neurons to TDP-43 pathogenicity.

In order to evaluate TDP-43 mis-localisation and aggregation, cortical neurons were transfected with a control (EGFP) construct, with a GFP-tagged TDP-43 wild-type (WT) construct, or with M337V or Q331K mutant constructs (here referred to as M and Q) and fixed at time points from 24 hours to 144 hours. Neurons were immunostained with anti-GFP antibodies to observe the distribution patterns of GFP control or TDP-43 isoforms. At all four time points, the GFP control protein was distributed through the entire neuron including axons and dendrites (Fig 1A–1D). At 24 and 48 hours, TDP-43 wild-type and mutant isoforms were strongly localised within the cell body, with weaker fluorescence along axons (Fig 1E, 1F, 1I, 1J, 1M and 1N). At 24 hours and t 48 h a lesser extent at 48 hours, TDP-43 WT axonal localisation as reflected by GFP fluorescence appeared slightly less than for the mutants (Fig 1E’, 1I’, 1M’, 1F’, 1J’, 1N’, 1H’, 1L’ and 1P’). By 72 hours, this differential was lost and fluorescence in the cell body and axons was equalised (Fig 1G, 1K, 1O, 1G’, 1K’ and 1O’). Cultures fixed at 96–144 hours showed an identical pattern (data not shown; Fig 1H, 1L, 1P, 1H’, 1L’ and 1P’).

**Fig 1:** TDP-43 is mislocalised in cortical neurons. Rat cortical neurons were transfected with GFP control (A—D), and GFP-tagged TDP-43 wild-type and mutant isoforms (E—P) and analysed at 24–144 hours (H). Immunostained with anti-GFP antibodies. Scale bar = 10 µm. Insets (E’–P’)—higher power views of the corresponding panels above, converted to black and white pixels. Scale bar = 10 µm.

As a control for the tagged TDP-43 distribution, neurons were immunostained for tyrosinated tubulin, which is distributed throughout the neuron. Tubulin staining was seen throughout neurons transfected with all constructs at 24–144 hour timepoints, showing an even distribution relative to GFP, and validating the changes in TDP-43 localisation that were observed (Fig 2A–2R, 2S–2U, 2Y–2A’ and 2E’–2G’).

**Fig 2:** Cytoskeletal integrity is compromised over time in cortical neurons. Rat cortical neurons were transfected with GFP control, or GFP-tagged TDP-43 wild-type and mutant isoforms as labelled and analysed at 24, 72 H and 144 H. Immunostaining with anti-GFP (green) and anti-tyrosinated tubulin (red) antibodies. Cellular fragmentation was observed at 144 H (bottom right panel). Scale bar = 10 µm.

Transfected neurons were next double-labelled with antibodies to GFP (green) and TDP-43 (red); the latter detected both the endogenous (rat) protein and the transfected (human) protein. At 24, 72 and 144 hours, TDP-43 protein was detected only in the nuclei of neurons transfected with the GFP control, as expected (Fig 3A–3F). At 24 hours for WT and mutant TDP-43 tranfections, the protein was present at a low level in axons (data not shown), whereas at 72 and 144 hours, TDP-43 protein distribution was increased in the axons (Fig 3G–3Z). However, both the GFP-tagged TDP-43 and the immunostained TDP-43 signal appeared grainy, suggesting that TDP-43 protein had aggregated in axons. At 144 hours, this granular appearance was similar for the wild-type and mutant-transfected neurons (Fig 3J–3Z, 3M, 3T and 3A'). For the majority of neurons, it does not appear that this phenomenon is due to axonal fragmentation as opposed to protein aggregation, as axons appeared intact based on anti-tubulin immunostaining (data not shown; Fig 2S–2U, 2Y–2A' and 2E'–2G').

**Fig 3:** TDP-43 mislocalisation visualised with anti-TDP-43 antibodies. Rat cortical neurons were transfected with GFP control, and GFP-tagged TDP-43 wild-type and mutant isoforms as labelled and analysed at 72 H and 144 H. Immunostaining with anti-GFP (green) and anti-TDP-43 antibodies (red). Scale bar– 10 µm. Insets—higher power views of corresponding panels to the left, stained with anti-TDP-43 antibodies. Scale bar = 10 µm.

We observed that in cultures from 72 hours onwards (data not shown) and particularly at 144 hours, a minority of neurons in the WT and mutant TDP-43 transfected cultures showed evidence of axonal disintegration and cell death. At 144 hours, dying or dead cells appeared as a series of spots, which were GFP-positive (reflecting TDP-43 localisation) and tubulin-positive (Fig 2V–2X, 2B'–2D' and 2H'–2J').

We have therefore shown that TDP-43 wild-type and mutant proteins were re re-distributed to axons over 0–72 hours, whereas at 144 hours, there is a suggestive appearance of aggregate formation, with evidence of neuronal fragmentation. However, fractionation assays have to be done to ascertain the nature of these aggregates. These data suggest that the mislocalisation of TDP-43 protein in cortical axons precedes neuronal disintegration.

### Over-expression of wild-type and mutant TDP-43 isoforms causes neurotoxicity in cortical neurons

We have previously shown that over-expression of the wild-type and mutant isoforms of TDP-43 causes neurotoxicity *in vivo* in chick embryo spinal cord [21]. In order to further investigate the cell death mentioned above, we quantitated neuronal cell death in cortical neurons using a TUNEL and a fluorometric cell viability assay, over 24–168 hours in culture. For the TUNEL assay, dead cells were counted manually at 24–72 hours (Fig 4A–4D). EGFP-expressing control neurons had few apoptotic cells at all three time points whereas the number of apoptotic cells was significantly higher for neurons expressing TDP-43 isoforms (Fig 4E). At 24–72 hour time points, the neurons over-expressing the wild-type and mutant isoforms of TDP-43 showed a significant increase in the number of apoptotic cells compared to the neurons expressing EGFP (* p < 0.01, ** p < 0.001, *** p < 0.0001; Fig 4E). There was no significant difference in toxicity between the TDP-43 wild-type and mutant constructs at each timepoint (p > 0.05). Overall, the numbers of apoptotic cells in TDP-43-transfected cultures were found to increase between 24 and 72 hours. In particular, the TDP-43 transfected cells showed a significant increase in cell death between 24 and 48 hours, and between 48 and 72 hours (* p < 0.01, ** p <0.001, *** p <0.0001: Fig 4E).

**Fig 4:** TDP-43 isoforms mediate toxicity in vitro. Control and TDP-43 transfected neurons (as labelled) were stained using a TUNEL kit and imaged to show TUNEL-positive cells (black dots) and Hoechst staining (white dots) after 72H in culture (A—D). Scale bar = 10 µm. (E) Average number of apoptotic cells quantified from five 0.24mm^2^ fields, at 3 time points as shown (3 experiments). Data is presented as means and standard errors. Significance was compared by ANOVA with GFP control at the respective timepoint and between constructs at various timepoints (no significance: p > 0.05; *** P < 0.0001, ** P < 0.001, * P < 0.01—compared with GFP control). (F) Semi-quantitative analysis of the viability of transfected cells assessed by Promega real-time glo viability assay at different time points from 3 experiments.

We also determined cell viability using a bioluminescent assay which is non-lytic and measures the metabolic activity of cells. We found that the GFP-transfected control cells showed greater viability than the TDP-43 transfected neurons at all timepoints, with an increase in cell numbers from 24–72 hours which likely reflects cell division in vitro (Fig 4F). There was a slight decrease in the viability of GFP-transfected cells between 72 and 168 hours in vitro, but overall, they showed a ~1.5 – 2x enhancement of viability relative to cells transfected with TDP-43 isoforms. All three TDP-43-transfected cell populations showed a decline in neuronal numbers between 72 and 168 hours (WT and M mutant) or 48 hours and 168 hours (Q mutant). These data suggest that the viability of neurons transfected with WT and mutant TDP-43 isoforms is significantly lower than for control cells, with the Q mutant showing the highest toxicity, and with an earlier onset. We conclude that TDP-43 isoforms cause a broadly similar level of toxicity in primary cortical neurons *in vitro*, with a slightly increased effect of the Q mutant construct.

### TDP-43 affects axonal growth and growth cone size *in vitro*

In order to characterize the effects of TDP-43 on cortical axon outgrowth, axon lengths were measured at 24–72 hours post-transfection after immunostaining with anti-GFP antibodies. Quantification suggested that control GFP-transfected neurons were longest at all time points whereas at 24 and 48 hours the TDP-43 transfected neurons (wild-type and mutants) show a modest reduction in neuronal length compared to the controls, which were significant at the p < 0.0001 level (Fig 5A). At 72 hours, it was surprising to note that the TDP-43 WT construct resulted in significantly shorter axons (p < 0.0001) relative to the control, whereas the mutant constructs produced only a modest reduction relative to the control (p < 0.05). Nevertheless, all three constructs impaired axon outgrowth in vitro.

**Fig 5:** TDP-43 affects axonal growth *in vitro*. (A) Quantitation of axon lengths of transfected neurons at time-points as labelled (n = 3 experiments; 100 neurons per experiment). Data is presented as means and standard errors. Significance were compared by ANOVA between constructs at same time points (no significance—p > 0.05; * P < 0.01; ** P < 0.001; *** P < 0.0001). (B)–(M) typical cortical neuron growth cones stained with anti-tyrosinated tubulin antibodies at timepoints and with constructs as labelled. Scale bar = 10 µm. (N) Quantitation of mean growth cone area at 3 different time points as labelled (70 neurons per construct per experiment, 3 experiments). Data is presented as mean and standard error. Significance denoted as for (A).

We noticed that some transfected cortical neurons had small growth cones, and quantitated this from 24–72 hours post-transfection by immunostaining with anti-GFP and anti-tubulin antibodies, and measuring growth cone areas (Fig 5B–5M). GFP-expressing control neurons have a characteristic ‘palm’ appearance with many filopodial extensions (Fig 5B, 5F and 5J). Growth cones of neurons transfected with TDP-43 constructs varied in morphology, but there was a trend for more spiky growth cones with smaller areas than GFP-transfected neurons. These difference were most pronounced at 72 hours, and both Q and M mutants affected growth cone morphology more strongly that WT-TDP-43 (Fig 5N and legend).

### TDP-43 affects axonal transport

The data obtained so far converge on the possibility that TDP-43 associates either directly or indirectly with proteins that affect cytoskeletal integrity, axonal outgrowth and growth cone dynamics. We next tested whether TDP-43 also affects anterograde transport of microtubule plus tip proteins, by studying the dynamics of EB3, a microtubule-associated protein that binds to the plus end of microtubules and regulates and promotes microtubule dynamics and growth [23]. Rat cortical neurons were co-transfected with GFP-tagged TDP-43 constructs and EB3-RFP and live imaged after 48 and 72 hours in culture. EB3 proteins, termed ‘comets’, move rapidly in an anterograde manner to the growing tips of axons (Fig 6A and 6A') and this movement can be analysed using kymographs.

**Fig 6:** TDP-43 affects anterograde transport in cortical neurons. (A) Example of a cortical neuron co-transfected with EB3-RFP, live imaged to show EB3 ‘comets’ (arrows) (A’) Higher power view. EB3 moves in an anterograde manner towards the growing ends of axon. (B)–(I) Example kymographs of neurons expressing GFP, or co-transfected with GFP and TDP isoforms, at 48 and 72H, as labelled. Distance along the X-axis and time along the Y-axis. Scale bar = 10 µm, except in A’ (J) Quantification of the velocity of EB3-RFP comets in the axons of transfected neurons. Graphs represent means and standard error of (n = 3). No significant differences were observed.

Kymographs show the tracks of EB3 comets, with the gradient of the tracks representing the velocity of movement (Fig 6B–6I). The kymographs show that the gradients for GFP controls are shallower than for TDP43-transfected neurons, and that the numbers of EB3 proteins are in general lower for the TDP M and Q mutants than for the EGFP control or the WT proteins. This suggests there may be fewer microtubules in TDP-Q-transfected cultures in particular, and that EB3 comets stop short of progressing to the ends of axons (Fig 6H and 6I). Quantitation of velocities show that there is trend towards the velocities being lower for TDP-43-transfected neurons than for controls; however these differences were not statistically significant (Fig 6J). This raises the possibility that TDP-43 can directly or indirectly impair axonal transport.

## Discussion

The aim of this study was to shed light on the mechanisms underlying TDP-43-mediated ALS. We have shown that TDP-43 mis-localises in cortical neurons and that the re-distribution is enhanced compared to that previously observed in spinal motor neurons [23]. Over-expression of TDP-43 wild-type and mutant proteins was toxic to cortical neurons and both mis-localisation and toxicity progressed with time. Rat cortical cells transfected with TDP-43 wild-type and mutant proteins showed varying phenotypes that reflected defective cytoskeletal functions; TDP-43 impairs axon outgrowth, microtubule and growth cone dynamics. Overall our results highlight the importance of cytoskeletal dysregulation as a factor in the pathophysiology of ALS. We have shown that axonal recruitment of TDP-43 begins at 24 hours and progresses with time, until at 144 hours, dying cells were observed in culture. Our findings are consistent with our previous studies using motor neurons in vitro and in vivo wherein TDP-43 showed progressive translocation from the nucleus into axons [21].

TDP-43 wild-type and mutant constructs were neurotoxic and the number of apoptotic cells increased over time, with the TDP-43 mutant Q331K showing the highest number of apoptotic cells across the different time points. The increased toxicity correlates with the progressive re-distribution of TDP-43. This is in accordance with several studies that show a positive correlation between TDP-43 toxicity and TDP-43 mislocalisation [24]. Comparatively, cellular fragmentation and toxicity was more severe in spinal motor neurons at 72 hours [21] whereas significant protein fragmentation was not observed until 144 hours in cortical neurons, suggesting that the former neuronal type may be more susceptible to TDP-43 aggregation.

A number of lines of evidence in this study showed that disruption of cytoskeletal integrity occurs in cortical neurons transfected with TDP-43 isoforms. TDP-43 transfected neurons showed a significant reduction in axon length, consistent with previous findings wherein over-expression of the TDP-43 WT caused a significant reduction in axon outgrowth in primary motor neurons when compared to the TDP-43 mutants [6]. TDP-43 transfected neurons also had smaller growth cones implying a defect in microtubule/actin dynamics. This was also reflected in the fragmentation of tubulin, implying that aggregation can lead to cell death by perturbing cytoskeletal integrity. We also report a trend towards decreased axonal transport.

Our results complement our previous findings in vivo wherein TDP-43 caused premature truncation and de-fasciculation of motor axons *in vivo* and reduced neurite outgrowth in chick spinal motor neurons *in vitro [21]*. The smaller growth cones we observe in this study could explain the shorter axons in vitro and the premature truncation and debundling/de-fasciculation of axons in vivo in chick spinal cord. It is plausible that growth cone defects could in turn lead to perturbations of axonal maintenance, which might contribute to neurodegeneration.

Axonal mRNA transport is considered to be a possible target of RNA-binding protein-mediated neurodegeneration and is a necessity for local translation [25]. Exome-wide rare variant analysis, identified patient variants of the tubulin alpha 4a (TUB4A) gene in familial ALS, thereby implicating the role of cytoskeletal defects in ALS [26]. We speculate that impairment in the mRNA regulation of TDP-43 binding partners may contribute to neurodegeneration via dysregulation of the axonal cytoskeleton.

The identification of mutations in several cytoskeletal genes in neurodegenerative diseases have highlighted their importance in the disease pathophysiology. Alzheimer’s disease, Parkinsons disease, Tauopathies, ALS, polyglutamine diseases all feature defects in cytoskeleton [27]. Cytoskeletal swellings, disruption of axonal transport and accumulation of cytoskeletal proteins in the abnormal inclusions are early events in neurodegeneration suggesting that disruption of the cytoskeleton initiates a cascade of events that eventually leads to atrophic processes.

## References

[1] NeumannM, SampathuDM, KwongLK, TruaxAC, MicsenyiMC, ChouTT, et al Ubiquitinated TDP-43 in frontotemporal lobar degeneration and amyotrophic lateral sclerosis. Science. 2006;314(5796):130–3. doi: 10.1126/science.1134108 1702365910.1126/science.1134108

[2] AraiT, HasegawaM, AkiyamaH, IkedaK, NonakaT, MoriH, et al TDP-43 is a component of ubiquitin-positive tau-negative inclusions in frontotemporal lobar degeneration and amyotrophic lateral sclerosis. Biochem Biophys Res Commun. 2006;351(3):602–11. doi: 10.1016/j.bbrc.2006.10.093 1708481510.1016/j.bbrc.2006.10.093

[3] KabashiE, ValdmanisPN, DionP, SpiegelmanD, McConkeyBJ, Vande VeldeC, et al TARDBP mutations in individuals with sporadic and familial amyotrophic lateral sclerosis. Nature genetics. 2008;40(5):572–4. doi: 10.1038/ng.132 1837290210.1038/ng.132

[4] SreedharanJ, BlairIP, TripathiVB, HuX, VanceC, RogeljB, et al TDP-43 mutations in familial and sporadic amyotrophic lateral sclerosis. Science. 2008;319(5870):1668–72. doi: 10.1126/science.1154584 1830904510.1126/science.1154584PMC7116650

[5] GitchoMA, BalohRH, ChakravertyS, MayoK, NortonJB, LevitchD, et al TDP‐43 A315T mutation in familial motor neuron disease. Annals of neurology. 2008;63(4):535–8. doi: 10.1002/ana.21344 1828869310.1002/ana.21344PMC2747362

[6] FalliniC, BassellGJ, RossollW. The ALS disease protein TDP-43 is actively transported in motor neuron axons and regulates axon outgrowth. Hum Mol Genet. 2012;21(16):3703–18. doi: 10.1093/hmg/dds205 2264181610.1093/hmg/dds205PMC3406762

[7] Van DeerlinVM, LeverenzJB, BekrisLM, BirdTD, YuanW, ElmanLB, et al TARDBP mutations in amyotrophic lateral sclerosis with TDP-43 neuropathology: a genetic and histopathological analysis. The Lancet Neurology. 2008;7(5):409–16. doi: 10.1016/S1474-4422(08)70071-1 1839610510.1016/S1474-4422(08)70071-1PMC3546119

[8] IgazLM, KwongLK, Chen-PlotkinA, WintonMJ, UngerTL, XuY, et al Expression of TDP-43 C-terminal fragments in vitro recapitulates pathological features of TDP-43 proteinopathies. Journal of Biological Chemistry. 2009;284(13):8516–24. doi: 10.1074/jbc.M809462200 1916428510.1074/jbc.M809462200PMC2659210

[9] VanceC, RogeljB, HortobágyiT, De VosKJ, NishimuraAL, SreedharanJ, et al Mutations in FUS, an RNA processing protein, cause familial amyotrophic lateral sclerosis type 6. Science. 2009;323(5918):1208–11. doi: 10.1126/science.1165942 1925162810.1126/science.1165942PMC4516382

[10] WegorzewskaI, BellS, CairnsNJ, MillerTM, BalohRH. TDP-43 mutant transgenic mice develop features of ALS and frontotemporal lobar degeneration. Proc Natl Acad Sci U S A. 2009;106(44):18809–14. doi: 10.1073/pnas.0908767106 1983386910.1073/pnas.0908767106PMC2762420

[11] Lagier-TourenneC, ClevelandDW. Rethinking ALS: the FUS about TDP-43. Cell. 2009;136(6):1001–4. doi: 10.1016/j.cell.2009.03.006 1930384410.1016/j.cell.2009.03.006PMC3110083

[12] AraiT, HasegawaM, AkiyamaH, IkedaK, NonakaT, MoriH, et al TDP-43 is a component of ubiquitin-positive tau-negative inclusions in frontotemporal lobar degeneration and amyotrophic lateral sclerosis. Biochemical and biophysical research communications. 2006;351(3):602–11. doi: 10.1016/j.bbrc.2006.10.093 1708481510.1016/j.bbrc.2006.10.093

[13] BurattiE, BaralleFE. The multiple roles of TDP-43 in pre-mRNA processing and gene expression regulation. RNA biology. 2010;7(4):420–9. 2063969310.4161/rna.7.4.12205

[14] TollerveyJR, CurkT, RogeljB, BrieseM, CeredaM, KayikciM, et al Characterizing the RNA targets and position-dependent splicing regulation by TDP-43. Nature neuroscience. 2011;14(4):452–8. doi: 10.1038/nn.2778 2135864010.1038/nn.2778PMC3108889

[15] StrongMJ, VolkeningK, HammondR, YangW, StrongW, Leystra-LantzC, et al TDP43 is a human low molecular weight neurofilament (hNFL) mRNA-binding protein. Mol Cell Neurosci. 2007;35(2):320–7. doi: 10.1016/j.mcn.2007.03.007 1748191610.1016/j.mcn.2007.03.007

[16] CoyneAN, SiddegowdaBB, EstesPS, JohannesmeyerJ, KovalikT, DanielSG, et al Futsch/MAP1B mRNA is a translational target of TDP-43 and is neuroprotective in a Drosophila model of amyotrophic lateral sclerosis. J Neurosci. 2014;34(48):15962–74. doi: 10.1523/JNEUROSCI.2526-14.2014 2542913810.1523/JNEUROSCI.2526-14.2014PMC4244467

[17] WangI-F, WuL-S, ShenCJ. TDP-43: an emerging new player in neurodegenerative diseases. Trends in molecular medicine. 2008;14(11):479–85. doi: 10.1016/j.molmed.2008.09.001 1892950810.1016/j.molmed.2008.09.001

[18] FieselFC, KahlePJ. TDP‐43 and FUS/TLS: cellular functions and implications for neurodegeneration. FEBS Journal. 2011;278(19):3550–68. doi: 10.1111/j.1742-4658.2011.08258.x 2177738910.1111/j.1742-4658.2011.08258.x

[19] WegorzewskaI, BalohRH. TDP-43-based animal models of neurodegeneration: new insights into ALS pathology and pathophysiology. Neurodegener Dis. 2011;8(4):262–74. doi: 10.1159/000321547 2112400410.1159/000321547PMC3214943

[20] BarmadaSJ, SkibinskiG, KorbE, RaoEJ, WuJY, FinkbeinerS. Cytoplasmic mislocalization of TDP-43 is toxic to neurons and enhanced by a mutation associated with familial amyotrophic lateral sclerosis. J Neurosci. 2010;30(2):639–49. doi: 10.1523/JNEUROSCI.4988-09.2010 2007152810.1523/JNEUROSCI.4988-09.2010PMC2821110

[21] TripathiVB, BaskaranP, ShawCE, GuthrieS. Tar DNA-binding protein-43 (TDP-43) regulates axon growth in vitro and in vivo. Neurobiol Dis. 2014;65:25–34. doi: 10.1016/j.nbd.2014.01.004 2442364710.1016/j.nbd.2014.01.004PMC3988849

[22] ArnoldES, LingS-C, HuelgaSC, Lagier-TourenneC, PolymenidouM, DitsworthD, et al ALS-linked TDP-43 mutations produce aberrant RNA splicing and adult-onset motor neuron disease without aggregation or loss of nuclear TDP-43. Proceedings of the National Academy of Sciences. 2013;110(8):E736–E45.10.1073/pnas.1222809110PMC358192223382207

[23] StraubeA, MerdesA. EB3 regulates microtubule dynamics at the cell cortex and is required for myoblast elongation and fusion. Current Biology. 2007;17(15):1318–25. doi: 10.1016/j.cub.2007.06.058 1765825610.1016/j.cub.2007.06.058PMC1971230

[24] BarmadaSJ, SerioA, ArjunA, BilicanB, DaubA, AndoDM, et al Autophagy induction enhances TDP43 turnover and survival in neuronal ALS models. Nature chemical biology. 2014;10(8):677–85. doi: 10.1038/nchembio.1563 2497423010.1038/nchembio.1563PMC4106236

[25] AlamiNH, SmithRB, CarrascoMA, WilliamsLA, WinbornCS, HanSS, et al Axonal transport of TDP-43 mRNA granules is impaired by ALS-causing mutations. Neuron. 2014;81(3):536–43. doi: 10.1016/j.neuron.2013.12.018 2450719110.1016/j.neuron.2013.12.018PMC3939050

[26] SmithBN, TicozziN, FalliniC, GkaziAS, ToppS, KennaKP, et al Exome-wide rare variant analysis identifies TUBA4A mutations associated with familial ALS. Neuron. 2014;84(2):324–31. doi: 10.1016/j.neuron.2014.09.027 2537435810.1016/j.neuron.2014.09.027PMC4521390

[27] McMurrayCT. Neurodegeneration: diseases of the cytoskeleton? Cell Death And Differentiation. 2000;7:861 doi: 10.1038/sj.cdd.4400764 1127953010.1038/sj.cdd.4400764

